# mRNA-Modified FUS/NRF2 Signalling Inhibits Ferroptosis and Promotes Prostate Cancer Growth

**DOI:** 10.1155/2022/8509626

**Published:** 2022-08-05

**Authors:** Ning Wang, Ying Yu, Rongjiang Wang, Yu Chen, Jianer Tang

**Affiliations:** ^1^Department of Urology, The First People's Hospital Affiliated to Huzhou Normal College, Huzhou 313000, China; ^2^Department of Surgery, The First People's Hospital Affiliated to Huzhou Normal College, Huzhou 313000, China

## Abstract

**Objective:**

Regarding the imperfect mechanism of occurrence and development of prostate adenocarcinoma (PRAD), this study investigated mRNA-modified FUS/NRF2 signalling to inhibit ferroptosis and promote prostate adenocarcinoma growth.

**Methods:**

Bioinformatics analysis was used to obtain the expression of FUS and its mRNA modification in PRAD. The expression of FUS in prostate cells (CRPC) and the level of m^6^A methylation modification, ferroptosis (P53 and GPX4), apoptosis (Caspase3), ferroptosis (P53 and GPX4), and apoptosis (Caspase3) in CRPC after ferroptosis inducer Erastin, ferroptosis inhibitor, and FUS knockdown were detected. Autophagy (LC3B), oxidative stress (GSH and ROS), and expression of NRF2/HO-1 pathway are indicators.

**Results:**

FUS was highly expressed in PRAD and phenomenally reduced the survival rate of patients. After knocking down FUS, the level of m^6^A methylation was significantly reduced, and the expressions of ferroptosis markers P53 and GPX4 were phenomenally reduced, while the levels of apoptosis and autophagy markers Caspase3 and LC3B remained unchanged. Upregulated and NRF2/HO-1 pathway indicators were upregulated. It shows that m^6^A methylation modification is reduced when FUS is the low expression, inhibits the expression of P53 and GPX4, downregulates GSH, upregulates ROS, activates the NRF2/HO-1 pathway, and promotes ferroptosis to inhibit the occurrence of RPAD.

**Conclusions:**

The increase of m^6^A methylation modification can increase the expression of FUS, thereby promoting the expression of P53 and GPX4, upregulating GSH, downregulating ROS, inhibiting the NRF2/HO-1 pathway, inhibiting ferroptosis, and promoting the growth of PRAD.

## 1. Introduction

Prostate adenocarcinoma (PRAD) is the most common tumor in men, with high morbidity and mortality [1, 2]. Surgery and chemotherapy are the main means of PRAD treatment, but the recurrence rate is high, and the prognosis is poor [3, 4]. Due to the limited treatment of PRAD contemporary, it is necessary to explore its pathogenesis and provide guidance for the early diagnosis and treatment of PRAD. Ferroptosis is a nonapoptotic or autophagy death mode caused by the accumulation of iron-dependent lipid peroxides [5–7]. Ferroptosis is involved in regulating the pathogenesis of various urinary tumors such as PRAD, bladder cancer, and kidney cancer [6]. The most common inducer of ferroptosis is Erastin, which activates multiple pathways quickly and persistently and is suppressed by the ferroptosis disease inhibitors Fer-1, DFO, and NAC [5, 6]. The induction of ferroptosis is related to the imbalance of oxidation level, involving excessive accumulation of reactive oxygen species (ROS) and release of oxygen free radicals, etc. [5–8]. At the same time, glutathione peroxidase 4 (GPX4) can inhibit peroxide under the action of glutathione (GSH), thereby inhibiting ferroptosis and promoting the growth of cancer cells [9, 10]. An NRF2 signalling pathway is closely related to ferroptosis, and NRF2 can bind with antioxidant elements to activate downstream HO-1 to regulate iron and ROS [11–15]. Therefore, exploring the mechanism of gene regulation of NRF2/HO-1 pathway is necessary to inhibit ferroptosis-induced PRAD.

The modification methods of mRNA consist of N6-adenine (m^6^A), n1-adenine (m1A), pseudouracil, and 5′-cytosine methylation, of which m6A is the most common [10, 16]. These modifications affect the splicing, expression, and translation of mRNA, etc. Previous studies have found that FUS, SMAD4, and DERL1 may be tumor markers by analyzing cancer samples from PRAD patients [17]. The fused sarcoma protein (FUS) is involved in the presplicesome of mRNA and gene transcription, etc. [1, 18]. Meanwhile, it was an important marker of PRAD occurrence and death [19]. Therefore, it was speculated that mRNA modified by the FUS might induce PRAD by regulating ferroptosis. This study mainly explored the mechanism by which mRNA modified gene expression regulation pathways participate in ferroptosis-induced PRAD, specifically, the mechanism by which m^6^A methylated FUS inhibits ferroptosis and promotes PRAD growth by regulating NRF2/HO-1 pathway. This study mainly examined FUS expression, m^6^A methylation modification level, ferroptosis index P53 and GPX4, apoptosis autophagy index Caspase3 and LC3B, oxidative stress index GSH and ROS, and NRF2/HO-1 pathway index expression. In order to provide a new idea for the pathogenesis of PRAD is conducive to the early diagnosis of PRAD, ameliorating the prognosis effect.

## 2. Material and Method

### 2.1. General Material

Prostate cancer cell lines RWPE-1, PC3, DU145, LNCaP, and C42 were purchased from American ATCC. DMEM culture medium is from Thermo Fisher; fetal bovine serum is from Gibco; RNA extraction kit, reverse transcription kit, and qPCR kit are from Shanghai Biyuntian; SiRNA and low expression FUS (shFUS) are from Shanghai; ferroptosis inducer Erastin, specific ferroptosis inhibitor FER-1, DFO, and NAC are from Selleck; glutathione (GSH) and reactive oxygen species (ROS) kits are from Nanjing.

### 2.2. Method

#### 2.2.1. Cell Culture and Transfection

The resuscitated prostate cancer cells RWPE-1, PC3, DU145, LNCaP, and C42 were cultured in a DMEM medium containing double antibodies (streptomycin/penicillin) and 10% fetal bovine serum, in which LNCaP cells were supplemented with NaHCO3 and pyruvate. The cell suspension was inoculated in a petri dish with appropriate density and then cultured in a 5%CO2 cell incubator at 37°C. After each cell line was stably cultured for 3 generations to form a stable cell line, it was communicated every two days for subsequent experimental studies. Among the different prostate cell lines selected, LNCaP and C42 cell lines had the highest expression of FUS and were consistent with the results of clinical samples, so LNCaP and C42 cell lines were selected for follow-up studies. LNCaP and C42 cell lines with low FUS expression were constructed after transfection with shFUS at a concentration of 150 nmol/*μ*l.

#### 2.2.2. MTT Detecting Cell Vitality

Among the different prostate cell lines selected, LNCaP and C42 cell lines had the highest expression of FUS and were consistent with the results of clinical samples, so LNCaP and C42 cell lines were selected for follow-up studies. LNCaP and C42 cells were cultured in 96-well plates and knocked down with the ferroptosis inducer Erastin, the ferroptosis inhibitor FRE-1, siRNA, and FUS, respectively. After the cells were grown for 48 hours, 20 *μ*L of MTT was added to each well, incubated for 3 to 4 h, discarded the culture medium, added 150 *μ*L DMSO, and shocked for 30 min. Check the OD value at 450 nm wavelength. Four replicate wells were set up in each group, and three replicate experiments were performed.

#### 2.2.3. GSH and ROS Detections

The LNCaP and C42 cell lines were selected for follow-up studies because they had the highest expression of FUS and were consistent with the clinical sample results. Consistent with previous experiments, LNCaP and C42 cells were seeded into 96-well plates and treated with Erastin, E + Fre − 1, siRNA, and FUS knockdown, respectively. After 48 h of incubation, wash with PBS and centrifuge. The cells were rapidly frozen and remelted by liquid nitrogen twice. Then, the cells were centrifuged, and the supernatant was taken for detection according to the instructions of the GSH and ROS kit, and the OD value was detected at 450 nm.

#### 2.2.4. Detection Index of qRT-PCR

qRT-PCR was performed by extracting total RNA from normal, Erastin, E + Fre − 1, siRNA, and shFUS treated LNCaP and C42 cells using TRIzol reagent to determine the concentration and purity of RNA. The RNA was then reversely transcribed into cDNA, and the mRNA levels of TLR4, MyD88, and NF-*κ*B were determined by quantitative fluorescence PCR. Reaction conditions are 95°C denaturation for 5 min, 94°C 30 s, 57°C 30 s, 72°C 30 s, 30 cycles, and 72°C extension for 5 min. Using GAPDH as an internal reference, the mRNA expression levels of each target were determined by the 2 − *ΔΔ*CT method. Primer sequences are shown in Table 1.

#### 2.2.5. Modification Level Detection of m^6^A

OligodT magnetic beads were used to extract siRNA and mRNA of shFUS treated LNCaP and C42 cells according to the kit, and the mRNA length was interrupted to 200 nt. Subsequently, the mRNA was incubated with antibodies and deliberately enriched, and 10% of RNA was isolated as input. Elution and reverse transcription of RNA eluted by m^6^A antibody, IgG antibody, and INPUT RNA were performed. PCR reaction used the designed m6A -IP-qPCR primers to detect the m6A modification level.

### 2.3. Statistical Method

SPSS 22.0 software was adapted for statistical data processing and analysis, the results were expressed as mean ± standard deviation, one-way ANOVA was used, and *P* < 0.05 was statistically phenomenal. GraphPad Prism 9 software is applied to visualize the results of statistical analysis. TCGA database was used for FUS expression level and biogenic prognosis analysis, and the RMBase V2.0 database was used to query FUS mRNA modification patterns.

## 3. Outcome

### 3.1. FUS Expression and Prognosis in Patients with PRAD

Using the TCGA database, it could be analyzed that FUS expression in patients with PRAD (497) and normal tissues (52) and found that FUS expression were phenomenally upregulated in patients with PRAD (*P* < 0.001) (Figure 1(a)). Analysis of survival curve results showed that the survival rate of patients with high FUS expression was phenomenally reduced, with *P* = 0.029 (Figure 1(b)). Subsequently, it was also analyzed that P53 activation and FUS expression and found that FUS expression were phenomenally higher in P53-activated PRAD patients (38 cases) than in normal controls and P53-inactive PRAD patients (*P* < 0.001) (Figure 1(c)). In conclusion, FUS expression is upregulated in PRAD patients, which phenomenally affects survival, and FUS expression is positively correlated with P53 activation.

### 3.2. FUS Expression in Different PRAD Cells

In order to better screen cell lines consistent with clinical results, we will select two cell lines with high FUS expression from the involved cell lines for follow-up studies. The mRNA expression levels of FUS in various prostate cells (CRPC) were detected, and it turned out that the FUS expression levels were RWPE-1, PC3, DU145, LNCaP, and C42 from low to high. FUS expression levels were phenomenally higher in other cells than in benign RWPE-1 (Figure 2(a)). Subsequently, LNCaP and C42 cells with relatively high FUS expression levels were selected for follow-up studies. Lentivirus infection was used to successfully construct LNCaP and C42 cell lines with low FUS expression, FUS expression rates were reduced by 80% to 90%, and the RNA transfection efficiency was 90% (Figures 2(b) and 2(c)). The results showed that FUS was also highly expressed in CRPC, with the most phenomenal difference between LNCaP and C42 cells.

### 3.3. Modification Detection of mRNA

In the early stage of the study, through querying the RMBase V2.0 database, it was found that the FUS mRNA modification mode was shown in Figure 3(a), m^6^A (91%) was the main mRNA modification mode, followed by 2′-O-Me (6%) and PseudoU (3%) (Figure 3(a)). Subsequently, the merIP-PCR assay was used to detect the methylation changes of mRNA m^6^A after FUS knockdown. Normalized treatment results showed that m^6^A methylation levels in the FUS knockdown group were phenomenally reduced (*P* < 0.01) in the same amount of RNA samples (200 ng, 100 ng, and 50 ng) of LNCaP and C42 cells (Figures 3(b) and 3(c)). In conclusion, m^6^A methylation is the dominant expression of FUS mRNA, and there is a positive correlation between FUS expression and m^6^A methylation.

### 3.4. Ferroptosis Model Construction and Index Detection

Previous studies have shown that 10 *μ*M Erastin treatment can induce ferroptosis in cells. Subsequently, ferroptosis inhibitors (FER-1 (1 *μ*M), DFO (100 *μ*M), and NAC (10 mm)) were added to observe the callback effect and ensure the successful construction of the model. As shown in Figures 4(a) and 4(b), cell viability was phenomenally alleviated after Erastin treatment (*P* < 0.01), but was reversed in the ferroptosis inhibitor group with no phenomenal difference compared with the control group (*P* > 0.05). Subsequently, we examined FUS expression in Erastin- and Fer-1-treated cells (Figures 4(c) and 4(d)) and found that Erastin was associated with downregulation of FUS expression, while FUS expression was reversed after Fer-1 treatment, showing no difference from the control group. These results indicated that ferroptosis that occurred in LNCaP and C42 cells was accompanied by downregulation of FUS expression, suggesting that high FUS expression may accelerate the occurrence and development of PRAD by inhibiting ferroptosis.

P53 and GPX4 were the key regulatory genes of ferroptosis, and the previous search of TCGA database found that FUS expression was phenomenally correlated with P53 activation in RPAD. Subsequently, it was detected the expression of P53 and GPX4 after ferroptosis inducer Erastin, ferroptosis inhibitor Fre-1, and FUS knockdown treatment. As shown in Figures 5(a) and 5(b), the expression of P53 was phenomenally alleviated in both LNCaP and C42 cells treated with Erastin and shFUS (*P* < 0.01) and reversed after the addition of the ferroptosis inhibitor FRE-1. Similarly, GPX4 expression was phenomenally downregulated after Erastin and shFUS treatment and reversed after the addition of FRE-1. This study further demonstrated that FUS high expression could inhibit ferroptosis and accelerate PRAD.

To further verify that FUS regulation of PRAD relies on cell ferroptosis rather than apoptosis or autophagy, the expression of apoptosis and autophagy markers Caspase3 and LC3B was examined after Erastin, E + FRE − 1, and FUS knockdown treatments. The results showed that Erastin, E + FRE − 1, and FUS knockdown treatments did not affect the expression of Caspase3 and LC3B in LNCaP and C42 cells (Figure 6), further demonstrating that FUS expression is related to the regulation of ferroptosis rather than apoptosis and autophagy.

### 3.5. Oxidative Stress Index Detection

Oxidative stress plays a crucial role in ferroptosis. The oxidative stress markers GSH and ROS expression were examined after Erastin, E + FRE − 1, and FUS knockdown treatments. Erastin was also used to construct the ferroptosis model, and the effect of a callback was observed by adding the inhibitor FRE-1. As shown in Figures 7(a) and 7(b), GSH expression was phenomenally downregulated after Erastin and shFUS treatment and phenomenally increased after Fre-1 supplementation, with no phenomenal difference from the normal group. ROS levels were phenomenally elevated after Erastin and shFUS treatment and reversed after Fre-1 supplementation (Figures 7(c) and 7(d)). These results suggest that FUS low expression can accelerate ferroptosis by downregulating GSH and upregulating ROS.

### 3.6. Pathway Indicator Detection of NRF2/HO-1

To further explore how FUS regulates ferroptosis-induced PRAD, NRF2/HO-1 pathway changes were examined after Erastin, E + FRE − 1, and FUS knockdown treatments. As shown in Figure 8, NRF2 and HO-1 expressions were phenomenally upregulated after Erastin and FUS knockdown treatments, whereas NRF2 and HO-1 expressions were phenomenally reversed after the supplemental inhibitor FRE-1 in ferroptosis model. These results suggest that FUS can induce PRAD by regulating the NRF2/HO-1 pathway to mediate ferroptosis.

In summary, FUS is highly expressed in PRAD and phenomenally reduces patient survival. After FUS knockdown, m^6^A methylation modification level was phenomenally reduced, and ferroptosis indicators P53 and GPX4 expression were phenomenally alleviated, while apoptosis and autophagy markers Caspase3 and LC3B levels were not changed, oxidative stress indicator GSH was downregulated, ROS was upregulated, and NRF2/HO-1 pathway was upregulated. These results suggest that FUS low expression can reduce m^6^A methylation modification, inhibit P53 and GPX4 expression, downregulate GSH, upregulate ROS, and activate NRF2/HO-1 pathway to accelerate ferroptosis and inhibit RPAD. In other words, increased m^6^A methylation and high FUS expression upregulate P53 and GPX4 levels, and downregulate the NRF2/HO-1 pathway to inhibit ferroptosis and accelerate PRAD.

## 4. Discussion

FUS is a member of the FET/TET protein family and is closely related to the pathogenesis of PRAD. Gleason pattern analysis also found that the frequency of FUS positive in nontumor tissues was lower than in PRAD tumor tissues [1]. Studies have found that low FUS expression in prostate cancer cell lines VCaP and LNCaP can phenomenally inhibit the expression of androgen AR and its downstream targets IGF1R and EGFR, thus inhibiting PRAD proliferation [19]. Other studies have found that FUS can combine with EMX2OS to synergistically activate the CGMP-PKG pathway to regulate the proliferation, migration, and invasion of CRPC [20]. In addition, FUS can interact with CIRC0005276 to activate XIAP and induce PRAD development [3]. This study shows that FUS is highly expressed in PRAD and CRPC, and low expression FUS PRAD has a higher survival rate.

A large number of previous studies have found that m^6^A methylation levels can regulate genes involved in the regulation of ferroptosis. Studies have found that m^6^A modification enhances ferroptosis in stellate cells by stabilizing BECN1mRNA to trigger autophagy activation [16]. Other studies have found that METTL3-mediated m^6^A methylation can stabilize SLC7A11mRNA and accelerate translation, thereby inhibiting ferroptosis and accelerating the proliferation of lung cancer cells [7]. In this study, we also found that increased m^6^A methylation levels upregulated FUS expression and inhibited ferroptosis.

Ferroptosis is the key link to induce PRAD. Erastin, a ferroptosis inducer, and second-generation antiandrogen RSL3 therapy phenomenally reduced CRPC growth and migration with no adverse effects [5]. OIP5-AS1 can regulate the expression of ferroptosis marker SLC7A11 through miR-128-3p, thus accelerating the progression of PRAD and ferroptosis resistance [7]. In addition, studies have found that flubendazole can induce P53 expression, downregulate ferroptosis markers SLC7A11 and GPX4 levels, and play an anti-CRPC proliferation and proapoptotic effect [9]. Similar to previous studies, this study found that FUS had low expression of ferroptosis indicators P53 and GPX4, while the levels of autophagy and apoptosis indicators Caspase3 and LC3B remained unchanged, accompanied by downregulation of oxidative stress factor GSH and upregulation of ROS. In conclusion, FUS inhibits ferroptosis and induces PRAD.

NRF2/HO-1 pathway is closely related to PRAD. Studies have found that PANX2 is highly expressed in PRAD, inhibiting ferrous and MDA levels and activating the NRF2/HO-1/FTH1 signalling pathway [21]. Other studies have found that P62 upregulates Nrf2 level and activity in PRAD and inhibits ROS by inhibiting KEAP1 [22]. Vitamin C and quercetin phenomenally downregulated Nrf2 expression levels in PC3 and DU145 cells, accompanied by alleviated oxidative stress indicators GPx, GR, and NQO1 enzyme activities [23]. In addition, other studies have found that low expression of PYGB in PRAD can regulate the expression of CASP3 and Bcl-2, upregulate ROS content, regulate the Nrf2 signalling pathway, and accelerate apoptosis of PC3 cells [24]. This study also found that ferroptosis was inhibited during FUS high expression, and the NRF2/HO-1 pathway was inhibited. These results suggest that low FUS expression in PRAD can accelerate ferroptosis induced by NRF2/HO-1 pathway.

In this study, the mechanism of increased m^6^A methylation accelerates FUS high expression and inhibits NRF2/HO-1 pathway to inhibit ferroptosis, accelerating PRAD at the cellular level. This mechanism will be further validated at a later stage. The specific regulatory mechanism in vivo will be verified by constructing a PRAD mouse model.

## 5. Conclusion

In summary, FUS is highly expressed in PRAD and phenomenally reduces patient survival. m^6^A methylation was phenomenally reduced in FUS low expression, and ferroptosis indicators P53 and GPX4 were downregulated, while the levels of autophagy and apoptosis indicators Caspase3 and LC3B remained unchanged, accompanied by downregulated GSH, upregulated ROS, and NRF2/HO-1 pathway activation. Conversely, increasing m^6^A methylation accelerates FUS high expression and inhibits NRF2/HO-1 pathway to inhibit ferroptosis, accelerating the occurrence of PRAD. This study provides a new idea of mRNA modification induction for the pathogenesis of PRAD, as well as the theoretical support for the early diagnosis and treatment of PRAD.

## Figures and Tables

**Figure 1:** FUS expression and prognosis in patients with PRAD. (a) Expression of normal tissue FUS in PRAD patients. (b) FUS expression and survival rate. (c) Relationship between FUS expression and P53 activation.

**Figure 2:** Different CRPC cells and FUS expression after knockdown. (a) FUS expression in different CRPC cells. (b) FUS expression in LNCaP cells after knockdown. (c) FUS expression in C42 cells after knockdown.

**Figure 3:** m^6^A methylation of FUS. (a) FUS mRNA modification type and proportion. (b) m^6^A methylation modification level in LNCaP cells. (c) Level of m^6^A methylation modification in C42 cells.

**Figure 4:** Effects of Erastin and ferroptosis inhibitor treatment on CRPC cell viability and FUS expression. (a) Cell viability of LNCaP cells after treatment. (b) Cell viability of C42 cells after treatment. (c) FUS expression of LNCaP cells after treatment. (d) FUS expression in C42 cells after treatment.

**Figure 5:** Effects of Erastin, ferroptosis inhibitor, and FUS knockdown on GPX4 and P53 expression. (a) P53 expression in LNCaP cells after treatment. (b) P53 expression in C42 cells after treatment. (c) GPX4 expression in LNCaP cells after treatment. (d) GPX4 expression in C42 cells after treatment.

**Figure 6:** Effects of Erastin, ferroptosis inhibitors, and FUS knockdown on Caspase3 and LC3B. (a) Caspase3 expression in LNCaP cells after treatment. (b) Caspase3 expression in C42 cells after treatment. (c) LC3B expression in LNCaP cells after treatment. (d) LC3B expression in C42 cells after treatment.

**Figure 7:** Effects of Erastin, ferroptosis rroptosis death inhibitors, and FUS knockdown on GSH and ROS. (a) GSH expression in LNCaP cells after treatment. (b) GSH expression in C42 cells after treatment. (c) ROS expression in LNCaP cells after treatment. (d) ROS expression in C42 cells after treatment.

**Figure 8:** Effects of Erastin, ferroptosis rroptosis death inhibitors, and FUS knockdown on NRF2 and HO-1. (a) NRF2 expression in LNCaP cells after treatment. (b) NRF2 expression in C42 cells after treatment. (c) HO-1 expression in LNCaP cells after treatment. (d) HO-1 expression in C42 cells after treatment.

**Table 1:** Primer sequences.

Primer	Upstream (5′-3′)	Downstream (5′-3′)
FUS	ATGGCCTCAAACGATTATACCCA	GTAACTCTGCTGTCCGTAGGG
shFUS	GAUUGGUAUUAUUAAGACATT	UGUCUUAAUAAUACCAAUCTT
P53	TTGAGGTGCGTGTTTGTG	CTGGGCATCCTTGAGTTC
GPX4	GAGGCAAGACCGAAGTAAACTAC	CCGAACTGGTTACACGGGAA
NRF2	ACACGGTCCACAGCTCATC	TGTCAATCAAATCCATGTCCTG
HO-1	AACTTTCAGAAGGGCCAGGT	CTGGGCTCTCCTTGTTGC
GAPDH	ACAGCCTCAAGATCATCAGC	GGTCATGAGTCCTTCCACGAT

## Data Availability

No data were used to support this study.
